# Genomic and Therapeutic Analyses of *Staphylococcus aureus* Isolated from Cattle Reproductive Tract

This article has been retracted.

**DOI:** 10.1155/2022/6240711

**Published:** 2022-09-13

**Authors:** Laiba Shafique, Amjad Islam Aqib, Qin Liang, Chaobin Qin, Muhammad Muddassir Ali, Memoona Adil, Zaeem Sarwar, Arslan Saleem, Muhammad Ajmal, Alveena Khan, Hongping Pan, Kuiqing Cui, Qingyou Liu

**Affiliations:** ^1^Guangdong Provincial Key Laboratory of Animal Molecular Design and Precise Breeding School of Life Science and Engineering, Foshan University, Foshan 528225, China; ^2^State Key Laboratory for Conservation and Utilization of Subtropical Agro-Bioresources, Guangxi University, Nanning, Guangxi 530005, China; ^3^Department of Medicine, Cholistan University of Veterianry and Animal Sciences, Bahawalpur 63100, Pakistan; ^4^Jinan City Zhangqiu District Animal Husbandry and Veterinary Development Center, China; ^5^Institute of Biochemistry and Biotechnology, University of Veterinary and Animal Sciences, Lahore 54000, Pakistan; ^6^Department of Theriogenology, Cholistan University of Veterinary and Animal Sciences, Bahawalpur-63100, Pakistan; ^7^Department of Aerospace and Geodesy, Technical University of Munich, Arcisstra. 21, 80333 Munich, Germany; ^8^Department of Veterinary Medicine, Sindh Agriculture University, Tandojam 70060, Pakistan; ^9^Allama Iqbal Medical College Lahore (University of Health Sciences), 54770, Pakistan

## Abstract

*Staphylococcus aureus* is emerging as a ubiquitous multidrug-resistant pathogen circulating among animals, humans, and their environment. The current study focused on molecular epidemiology and evidence-based treatment against *S. aureus* from bovine endometritis. For this study, *n* = 304 cattle were screened for endometritis using ultrasonography while presenting case history, and clinical signs were also considered. *S. aureus* was isolated from endometritis-positive uterine samples which were further put to molecular identification, phylogenetic analysis, susceptibility to antibiotics, and testing of novel drug combinations in both *in vitro* and field trials. The findings of the study revealed 78.20% of bovine endometritis samples positive for *S. aureus*, while *nuc* gene-based genotyping of *S. aureus* thermal nuclease (SA-1, SA-2, and SA-3) showed close relatedness with *S. aureus* thermal nuclease of *Bos taurus*. Drug combinations showed 5.00 to 188.88% rise in zones of inhibitions (ZOI) for drugs used in combination compared to the drugs used alone. Gentamicin in combination with amoxicillin and enrofloxacin with metronidazol showed synergistic interactions in an *in vitro* trial. Co-amoxiclav with gentamicin, gentamicin with enrofloxacin, and metronidazole with enrofloxacin showed 100%, 80%, and 60% efficacy in treating clinical cases in field trials, respectively. As a result, the study came to the conclusion the higher prevalence of endometritis-based *S. aureus*, genetic host shifts, narrow options for single drugs, and need for novel drug combinations to treat clinical cases.

## 1. Introduction

Endometritis is among the leading causes of morbidity in animals thus significantly compromising the farm economy [1, 2]. Reproductive manipulations around parturition are the principal source of bacterial invasions, resulting in severe uterine infections associated with huge economic losses compromising herd health and production [1]. Economic losses in terms of decreased reproductive efficiency, treatment costs, premature culling, increased services per conception, and pathogen transmission risks proclaim endometritis as one of the prime challenges in the dairy industry [2, 3]. Inflammatory expressions of the endometrium depict the fate of animals, as compromised fertility leads to premature culling [4]. *S. aureus* transfers at an animal-human-environment interface, thus making it a major threat to optimum reproductive efficiency in farm animals too [5–7]. Authentic diagnosis of various strains demands genome analyses because conventional microbiological methods are no longer enough [8]. It is noted that among several major challenges to the dairy farming industry is the drug resistance which presents itself as an invariably significant risk factor [9]. Resistance to commonly used antibiotics in animal-originated *S. aureus* isolates poses a threat to global public health [3, 10]. These strains commonly colonize mucosal surfaces and sustain their colonies by producing biofilm [7]. Drug resistance, localization in epithelium, longer attachment duration, bypassing immunity, and enhancement of pathogenesis make *S. aureus* a specific pathogen [11–13]. Some strains are also emerging as multidrug-resistant, even depicting reduced susceptibility to vancomycin [14]. MRSA is a salient contagious pathogen which is equally found in humans and animals [15]. According to the literature, the prevalence of MRSA varies from 0.4 percent in Hungary to 47.6 percent in China [16, 17].

To ensure optimum reproductive performance, it is necessary to combat *S. aureus*-based endometritis in dairy animals. Non-judicious exposure to antibiotics results in the development of resistance to pathogens. Certain antibiotics can act as antimicrobial signaling molecules, homeostatic modulators, and induce the transcription of virulent genes at sublethal levels [18]. Subminimal inhibitory concentration (sub-MIC) of drugs is unable to kill resistant bacteria but leads to modification of chemical and physical characteristics of the cell surface, adhesion mechanisms, and expressions of some of the virulent genes leading to biofilm formation, toxin production, motility, and 68 hydrophobicity [19, 20]. Approaches such as double antibiotic combination therapy has been suggested for the treatment of resistant *S. aureus* strains [21, 22]. Moreover, more efficacious antimicrobials are being sought to reduce the use of unnecessary medication. Thus, the hypothesis of the study reads “*Staphylococcus aureus* endometritis is prevalent in dairy animals, host shifts exist, and novel antibiotic combinations are effective against multidrug-resistant *S. aureus* isolates.”

## 2. Materials and Methods

### 2.1. Ethics Statement

This study was approved by the Experimental Animal Care and Use Committee of Guangxi University (No. GXU-2021-128 and dated 30-6-2020).

### 2.2. Tracking Endometritis Cases from Bovines

The study was conducted in selected dairy farms of the district of Khanewal, Punjab, Pakistan (Figure 1). District Khanewal is located at 71°55′0^″^E and 30°18′0^″^N with an altitude of 128 meters and a human population of 2.922 million. Clinical reproductive complaints were defined as any kind of reproductive problem, e.g., repeat breeding, abortion, misconception, and signs associated with these issues. The inclusion criteria for the current study were commercial dairy farms having ≥50 lactating cattle/farm, farm accessibility, reproductive complaints, and ultrasonographic findings. Supplementary information included calving history, milk yield/day, days in milk, parity, feeding regime, and treatment approach. Random sampling was done to check for endometritis in *n* = 304 cattle using ultrasonography (7.5 MHz with probe linear array transrectal; B mode) [23]. Endometritis was defined as a swollen lumen partly filled with snowy echogenic patches and black nonechogenic fluid [24, 25]. It was found that if all rays were reflected after striking any structure, the area looked whitish [26]. Clinical identification of animals having endometritis through ultrasonography is represented in Figure 2.

Aseptically, the uterine flushing was done by an artificial insemination gun whereas the fluid was taken out and stored by a syringe. The samples were shifted to the laboratory (central diagnostic laboratory) of CUVAS, Bahawalpur, Pakistan, in a container having 4°C temperature.

### 2.3. Isolation of Pathogenic *S. aureus*

The samples were put to incubation in sterile nutrient broth overnight at 37°C to retrieve the maximum yield of those bacteria which were present in a low quantity. The incubated nutrient broth was centrifuged, and the sediments were put to blood agar for the same incubation [27]. The colonies obtained were further put on Mannitol salt agar with the same incubation and preceded further to several biochemical tests as per set protocols [28].

### 2.4. Molecular Identification of Pathogenic *S. aureus*

Isolates biochemically characterized were further put to genomic analysis. PCR amplification was done with *Nuc* gene (Figure 3). Primers were formulated using Primer-BLAST (https://www.ncbi.nlm.nih.gov/tools/primer-blast/) software (Nuc forward 5′AAGGGCAATACGCAAAGAG3′ and Nuc reverse 5′AAACATAAGCAACTTTAGCCAAG3′) (figure reaction mixture consists of PCR 2X master mix = 10 *μ*L (Thermo Scientific Catalog #K0171), forward primer = 1 *μ*L (10 pmoL), reverse primer = 1 *μ*L (10 pmoL), DNA = 2 *μ*L (50 ng/L), deionized water = 6 *μ*L, and reaction volume = 20 *μ*L). The detailed protocol has been described in Aziz et al. [7].

### 2.5. Sequence Analysis of the Local *S. aureus* Isolate

A phylogenetic analysis of nucleotides was carried out with MEGA X software. Highly similar sequences acquired via Primer-BLAST were combined in a phylogenetic analysis of nucleotides of the *Nuc* gene in *S. aureus*. The phylogenetic tree was made to find lengths of branches in similar units like those of the evolutionary distances utilized to conclude the phylogenetic tree. Further, the maximum composite likelihood method was applied to find distances in the evolutionary tree, and the similar was calculated in unit numbers of substitutions of base pairs at each site. The rest of the protocol was done the same as described in the author's previous study (doi:10.3390/antibiotics10080997). Moreover, motifs were found through the MEME (Multiple EM for Motif Elicitation) Suite and STRING was used to find the protein-protein interaction.

### 2.6. Confirmation of Pathogenic Nature of *Staphylococcus aureus*

Using the cefoxitin disc diffusion assay [29], methicillin resistance in *S. aureus* was determined as per standards provided in clinical and laboratory standard institute [30]. Antibiotic discs were placed on Mueller Hinton agar on which *S. aureus* was already swabbed. Plates were incubated for 24 hours while zones of inhibition were measured and compared as per guidelines of the clinical and laboratory standard institute [30].

### 2.7. Molecular Confirmation of Methicillin-Resistant *Staphylococcus aureus*

The molecular confirmation of methicillin resistant *S. aureus* was done by targeting the *mecA* gene. DNA extraction was done by WizPrep™ gDNA Mini extraction kit. Amplification was done utilizing *mecA* forward P1: 59-TGGCATTCGTGTCACAATCG-39 and reverse primers P2: 59-CTGGAACTTGTTGAGCAGAG-3′ with amplified product size 310 bp as described by Shoaib et al. [31]. Further specification of PCR was followed by previously established protocol for identification of MRSA by targeting *mecA* in *S. aureus*. Bands examined at a 310 bp level were taken into consideration as positive (Figure 4).

### 2.8. Assessment of Antibiotic Resistance Profile of Methicillin-Resistant *Staphylococcus aureus*

Using the disc diffusion method, commonly used antibiotics were tested against drug-resistant *S. aureus* isolates according to the guidelines of clinical and laboratory standard institute [30]. The antibiotics tested were enrofloxacin (10 *μ*g), gentamicin (10 *μ*g), linezolid (30 *μ*g), vancomycin (30 *μ*g), trimethoprim-sulphamethoxazole (25 *μ*g), fusidic acid (10 *μ*g), ciprofloxacin (5 *μ*g), chloramphenicol (30 *μ*g), and levofloxacin (5 *μ*g). Antibiotics were aseptically placed on Mueller Hinton agar having swabbed with *S. aureus* and put to incubation for 24 hours at 37°C. The zone of inhibition of each antibiotic was measured and compared as per guidelines of the clinical laboratory and standard institute [30].

### 2.9. Synergy Testing of Novel Drug Combinations against MRSA

To validate the synergism of novel drug combinations, various drug combinations were tested using the agar and broth dilution methods [32]. To conduct well diffusion assay, 6–8 mm diameter wells were made through good borer on Mueller Hinton which was later swabbed with activated growth of bacteria [32]. To evaluate the antibacterial potential of the antibiotics, following drugs were used alone and in combination against *S. aureus*: amoxicillin, oxytetracycline, gentamicin, streptomycin, metronidazole, enrofloxacin, and co-amoxiclav. Zones formed around antibiotics were measured post-incubation. The checkerboard method was applied to find synergism between different combinations of drugs using broth microdilution protocol. An activated growth of *S. aureus* adjusted at 1–1.5 × 10^5^ *CFU*/*mL* was used in this trial. Optical density was calculated at 570 nm following incubation at 37°C/24 hours. Fractional inhibitory concentration indices (FICI) were calculated as per the following formula. Experiment was executed in triplicate [32].

(1) $$\begin{array}{c} \text{Fractional inhibitory concentration index}=\text{FIC product }A+\text{FIC product }B,\\ \text{FIC of Product }B=\frac{\text{MIC of Product }B\text{ in combination with Product }A}{\text{MIC of Product }B\text{ alone}},\\ \text{FIC of Product }A=\frac{\text{MIC of Product }A\text{ in combination with Product }B}{\text{MIC of Product }A\text{ alone}}. \end{array}$$

The fractional inhibitory concentration indices (FICI) ≤ 0.5 were considered as synergistic, FICI > 0.5 but ≤1.0 as additive, FICI > 1.0 but <4.0 as indifferent, and FICI > 4.0 considered as antagonistic [33].

### 2.10. Field Trial to Treat Endometritis

*Methicillin resistant S. aureus*positive endometritis cases were included in a field trial of drugs. Drugs selected for the trials were gentamicin, oxytetracycline, co-amoxiclav, amoxicillin, streptomycin, metronidazole, and enrofloxacin. The dosage regimen and drug combinations were as follows (Supplementary Table 1). The rate of success was calculated using the following criteria: (i) ultrasonography determined normal uterine walls, (ii) absence of bacterial load from vaginal/uterine discharge, and/or (iii) successful conception [34, 35]. The first two points were considered necessary while the third was kept optional because there might be other reasons for no conception.

### 2.11. Statistical Analysis

A univariate analysis was applied to the prevalence and antibiotic susceptibility [23]. An increase of percentage (%) in inhibition zones as well as in fractional inhibitory indices was computed by using formulae described previously [32, 33]. Parametric tests (ANOVA and *t*-tests) were applied for quantitative data. Tukey test was applied as post hoc test, a succession to ANOVA, to decide significant difference among groups at a 5% level of probability. SPSS version 22 of statistical computer software program was used for data analysis.

## 3. Results

### 3.1. Prevalence and Risk Factors Associated with *S. aureus*

The study showed 78.20% of endometritis samples positive for *S. aureus*, while 26.92% of these were MRSA (Table 1). Calving history, milk yield, days in milk, treatment approach, and feeding regimen were non-significant while parity showed significant (*p* < 0.05) association (Table 2).

### 3.2. Sequencing of *Staphylococcus aureus*

#### 3.2.1. Nucleotide Output

Nucleic acid alignment revealed that reference sequence and local isolate *S. aureus* thermal nuclease (SA-1, SA-2, and SA-3) sequences were found 99.8% identical (Supplementary Figure 1).

#### 3.2.2. Phylogenetic Analysis

According to constructed phylogenetic tree of *S. aureus thermal nuclease*, it was found that local isolate (SA-1, SA-2, and SA-3) gene sequence was closely linked to the *S. aureus thermal nuclease* of *Bos taurus* and from other bovine milk (Figure 5).

#### 3.2.3. Assessment of Motif and Structure of Gene

The nucleic acid motif of the reference sequence and all local isolates was found 1.13*e*-126. The differences in motifs were shown in different colors (Supplementary Figure 2). It was found that the coding region was only associated with nucleotide structure (Supplementary Figure 3). Protein motif of reference sequence and all local isolates was found 1.59*e*-172 (Figure 6(a)). Protein structure of reference protein and local isolate (SA-1, SA-2, and SA-3) proteins was found identical (Figure 6(b)). Protein motif *p* value of reference sequence and all local isolates was found (Figure 6(c)). Protein-protein interaction (Figure 6(d)) was noted in SA-1, SA-2, and SA-3 proteins. Conserved domain of the *Staphylococcal* nuclease was found in reference, Sample-1, Sample-2, and Sample-3 protein sequences (Supplementary Table 2).

### 3.3. Antibiogram against MRSA

An antibiogram of tested isolates showed trimethoprim-sulphamethoxazole and ciprofloxacin as highly effective antibiotics, while fusidic acid remained the least effective. The susceptibility profile of *S. aureus* against different antibiotics with “increasing number of resistant isolates” was observed as follows: trimethoprim-sulphamethoxazole > ciprofloxacin ≥ enrofloxacin ≥ chloramphenicol > gentamicin > levofloxacin > linezolid > vancomycin > fusidic acid (Figure 7). The antibacterial activity of different antibiotics represented by ZOIs can be seen in Supplementary Figure 4(i).

### 3.4. *In Vitro* Drug Synergy Testing

#### 3.4.1. Zone of Inhibition Expressed by Tested Drugs

The study revealed that metronidazole+gentamicin when compared with other drugs showed a significant difference (*p* < 0.05) of ZOIs (Table 3, Supplementary Figure 4ii). Drug combination analysis of well diffusion zones showed that there was a maximum increase in inhibitory zone for the combination of oxytetracycline with streptomycin when compared to oxytetracycline alone. The highest combination of drugs favored oxytetracycline in that there was more than a 100% increase in its ZOIs when combined with other drugs. Amoxicillin and enrofloxacin gave greater percentage increase when combined with gentamicin and chloramphenicol, respectively.

#### 3.4.2. Fractional Inhibitory Concentration Indices

The minimum inhibitory concentrations of all tested drugs varied significantly from each other. The lowest MIC was noted in the case of enrofloxacin which was followed by gentamicin, co-amoxiclav, amoxicillin, oxytetracycline, streptomycin, and metronidazole. Synergy testing of all the tested drug combinations against MRSA isolates showed synergistic behavior of amoxicillin+gentamicin and metronidazole+enrofloxacin, while antagonism was observed in oxytetracycline+amoxicillin and co-amoxiclav+oxytetracycline. An additive effect was found when amoxicillin was combined with enrofloxacin and streptomycin; co-amoxiclav with enrofloxacin and gentamicin; and enrofloxacin with gentamicin. All other remaining combinations remained indifferent (Table 4).

### 3.5. Field Trial Outcomes

The study noted the highest percentage recovery in case of co-amoxiclav+gentamicin, oxytetracycline alone, gentamicin+enrofloxacin, gentamicin alone, and metronidazole+enrofloxacin combinations presenting 100%, 100%, 80%, 80%, and 60% success rate, respectively. The uterine wall exhibiting normalization is shown in Figure 8. Amoxicillin+gentamicin, amoxicillin+streptomycin, and metronidazole+amoxicillin, on the other hand, showed success rates of 30%, 20%, and 10% against MRSA, respectively.

## 4. Discussion

The prevalence of *S. aureus* in this study was in line with previous studies in that aborted cattle revealed 17.2% endometritis and 88.3% *S. aureus* [36]. Different studies have also found that the number of people with MRSA seems to be lower (16.7% in Germany, 13.1% in India, and 4% in the USA), and the low expression of the *mecA* gene could be the cause of the varying outcomes for MRSA. The risk factors' association in our study was in agreement with results of a previous study [37]. Favorable climatic conditions and the presence of predisposing risk factors trigger the process of acquired resistance.

After the confirmation of phenotypical methods, the genomic confirmation of *S. aureus* with PCR is a reliable tool for the identification of species [8]. Other scientists also used the *nuc* gene to identify *S. aureus* [38, 39]. The MEME Suite web server is used for sequence analysis that provides information on protein interaction domains and DNA binding sites [40]. Gene structure servers provide gene images that describe gene structure and features. These, in turn, are required to further investigate evolution and functional attributes [41]. Different softwares are used for the identification of structural similarities that to some extent can be used to find functional attributes [42].

The vancomycin resistance reported in the present study resemble with the previous studies. This may be because of acquired resistance, as reported in the methicillin case [43]. Vancomycin resistance in *S. aureus* may also be because of acquired transposon Tn1546, via vancomycin-resistant *Enterococcus faecalis*, resulting from variations in the structure of the cell wall and cellular metabolism of isolates [44]. The study showed downward receptivity trends to enhanced penicillin that could be because of genetic variation in penicillin-binding proteins. Mutation in penicillin-binding proteins is proposed to change the capacity of antibiotics to the receptor proteins, resulting in an increasing MIC of penicillin group [29–31] and thus supports the findings of the current study. A similar pattern of MIC for commonly used drugs was reported in previous studies [45–48] against animal and human associated *S. aureus*. Sanganyado and Gwenzi [49] found that *tet* (A, B, C, G, O) and *tet* (W) genes which code for tetracycline resistance may be linked to higher MIC values for oxytetracycline. Streptomycin's MIC in the current study was in line with results reported by Zhang et al. [50], which showed that microbes have acquired resistant genes against streptomycin resulting in higher MIC values. Studies that evaluated milk samples have shown that *S. aureus* is resistant to multiple antibiotics in the same way [51].

Drug combination therapy for the treatment of MRSA infections is highly regarded in literature to avoid further resistance and to immediately clear the infection. Previous studies [32, 33, 52] found antimicrobial resistance to be tackled by combination of antibiotics with non-steroidal anti-inflammatory drugs. Similarly, plant extracts [53, 54] and nanoparticles [55, 56] were well documented with promising antimicrobial results. Changes in the results of the response to the drugs tested *in vivo* and *in vitro* agreed with previous studies [57–60]. The differences in the results could be attributed to binding pathways at cellular level, temperature changes, the effect of cellular matrix on drug activity [57], response of the immune system, enzymatic degradation [59], and pharmacokinetic and pharmacodynamic specifications of the living being [58]. These associated attributes make it hard to get reproducibility and similarity in results [61]. Rise in antimicrobial resistance with respect to novel strains like vancomycin resistant *S. aureus* [62] and presence of MRSAs not only in dairy udder [63] but also in companion livestock e.g poultry [64, 65] adds additional burden to the economy and health of animals as well as public.

## 5. Conclusion

The study confers hiked percentages of *S. aureus* in endometritis and found a clue of pathogen transfer from other animals. *In vitro* drug combinations showed many folds of antibacterial activity with very limited antagonism. In the field trials, novel drug combinations provided a wider range of treatment options which encouraged the use of evidence-based therapeutics instead of conventional treatment. It is therefore suggested that molecular epidemiology and evidence-based drug combinations should be regularly observed to culminate drug resistance and to save one's health.

## Figures and Tables

**Figure 1:** Tracking burden of (a) *S. aureus* from endometritis and (b) MRSA from different dairy farms (each circle is showing one dairy farm). In the second map (b) there are 9 farms as one farm in the first map (a) did not show *S. aureus*.

**Figure 2:** Clinical identification of animals having endometritis through (a, b) ultrasonography and (c) abnormal secretions. (a) EL = endometrial lining; E = endometritis in the form of swelling of the lining; PM = pus material; (b) EL = endometrial lining; E = endometritis in the form of an inflamed wall; (c) red arrows point out pus material from uterine material.

**Figure 3:** Molecular identification of *S. aureus*. M = marker 1000 bp; +VE = positive control wells 1–8 samples.

**Figure 4:** Molecular identification of methicillin-resistant *S. aureus*. M = marker leader 1000 bp, 1–9 wells were samples at 310 bp; positive control = +ve; negative control = −ve.

**Figure 5:** Phylogenetic tree of *S. aureus Nuc* gene (nucleotide sequences). An analysis has been performed among different source samples of *S. aureus Nuc* gene from different countries with our isolated sequenced samples. The branch length (numbers) is representing the nucleotide substitutions per 100 nucleotide sites.

**Figure 6:** (a) Protein structure (exonic region) of *S. aureus*. (b) Alignment of *S. aureus* thermal nuclease protein (*S. aureus*-1, *S. aureus*-2, *S. aureus*-3, and reference sequence). (c) Protein motifs of *S. aureus*. (d) Protein-protein interaction of *S. aureus* protein (*S. aureus*-1 protein, *S. aureus*-2 protein, and *S. aureus*-3 protein).

**Figure 7:** Antibiogram of *S. aureus* isolates. FA = fusidic acid; Enro = enrofloxacin; Cip = ciprofloxacin; TS = trimethoprim-sulphamethoxazole; Levo = levofloxacin; Chlor = chloramphenicol; Van = vancomycin; Gent = gentamicin; Line = linezolid.

**Figure 8:** Parameters of successful treatment and post treatment successful pregnancy: (a) normal endometrial lining (EL), (b) normal uterine secretions—clear string formed without any pus material, and (c) pregnancy established in animals as evident by developing.

**Table 1:** The prevalence of *Staphylococcus aureus* and methicillin-resistant *Staphylococcus aureus*.

Farm name	Prevalence of endometritis				*S. aureus* (%)			MRSA (%)		
	No. of animals screened	Endometritis positive	Prevalence	Confidence interval	*S. aureus* positive	*S. aureus*%	Confidence interval	MRSA positive	MRSA	Confidence interval
	(A)	(B)	(*B*/*A* × 100)	-95%	(C)	(*C*/*B* × 100)	-95%	(D)	(*D*/*C* × 100)	-95%
(A)	27	9	33.33	18.64-52.17	5	55.55	26.67-81.13	2	40	11.76–76.93
(B)	27	8	29.63	15.85–48.48	8	100	67.56–100	1	12.5	2.24–47.09
(C)	18	8	44.44	24.56–66.28	4	50	21.52–78.48	0	0	—
(D)	34	14	41.18	26.37–57.78	14	100	78.47–100	6	42.86	21.38–67.41
(E)	54	26	48.15	35.4–61.15	24	92.31	75.86–97.87	7	29.17	14.92–49.17
(F)	12	5	41.67	19.33–68.05	3	60	23.07–88.24	1	33.33	6.15–79.23
(G)	28	13	46.43	29.53–64.19	10	76.92	49.74–91.82	1	10	1.79–40.41
(H)	48	26	54.17	40.29–67.43	20	76.92	57.95–88.96	6	30	14.55–5.19
(I)	38	16	42.10	27.86–57.81	16	100	80.64–100	4	25	10.98–4.15
(J)	18	8	44.44	24.56–66.28	0	0	0.00–32.44	0	0	—
**Total**	304	133	**43.75**		104	78.20		28	26.92	

**Table 2:** Risk factors associated with methicillin-resistant *S. aureus* isolated from bovine endometritis.

Parameter	Categories	Total	Positive	% age	*p* value
Calving history	Dystocia	81	18	22.22	0.879
	Abortion	4	1	25	
	Eutocia	48	9	18.75	

Milk yield/day	10–20	38	8	21.05	0.956
	21–30	56	12	21.42	
	31–40	26	6	23.07	
	41–50	13	2	15.38	

Days in milk	1–100	86	19	22.09	0.919
	101–200	32	6	18.75	
	201–300	15	3	20	

Parity	1–3	76	21	27.63	0.032
	4–6	57	7	12.28	

Feeding regime	Silage+concentrate	43	10	23.25	0.832
	Silage+hay+concentrate	56	12	21.42	
	Silage+concentrate+fresh fodder	34	6	17.64	

Treatment approach	Single antibiotic	85	18	21.17	0.835
	Combination	48	10	20.83	

**Table 3:** Comparison of zones of inhibition against methicillin-resistant *Staphylococcus aureus* isolates using the well diffusion method for antimicrobial drugs alone and/or in combination.

Drugs	Patterns used (alone/combination)	Mean ± Std. (mm)	% variation [(combination-alone)/(alone×100)]	*p* value
Co-amoxiclav	Alone	15 ± 1.414		0.299
	C+E	12.5 ± 4.949	-16.67	
	C+M	11.5 ± 0.707	-23.33	
	C+G	10.5 ± 2.121	-30	
	C+O	9.5 ± 0.707	-36.67	
	C+A	10.5 ± 2.121	-30	
	C+S	9.0 ± 1.414	-40	

Enrofloxacin	Alone	6.0 ± 0		0.082
	E+M	5.5 ± 0.707	-8.33	
	E+G	4.5 ± 0.707	-25	
	E+O	7.5 ± 0.707	25	
	C+E	12.5 ± 4.949	108.33	
	E+A	10.0 ± 2.828	66.66	
	E+S	9.0 ± 1.414	33.33	

Metronidazole	Alone	6.0 ± 1.414		0.025
	M+G	8.5 ± 0.707	41.67	
	M+O	8.5 ± 0.707	41.67	
	C+M	11.5 ± 0.707	91.67	
	E+M	5.5 ± 0.707	-8.33	
	M+A	8.0 ± 1.414	33.33	
	M+S	7.5 ± 2.121	25	

Oxytetracycline	Alone	4.5 ± 0.707		0.093
	C+O	9.5 ± 0.707	111.11	
	M+O	8.5 ± 0.707	88.89	
	E+O	7.5 ± 0.707	66.67	
	G+O	9.5 ± 0.707	111.11	
	O+A	10.5 ± 3.535	133.33	
	O+S	13.0 ± 4.242	188.88	

Gentamicin	Alone	10 ± 2.828		0.034
	G+O	9.5 ± 0.707	-5	
	C+G	10.5 ± 2.121	5	
	E+G	4.5 ± 0.707	-55	
	M+G	8.5 ± 0.707	-15	
	G+A	16.0 ± 2.828	60	
	G+S	13.0 ± 4.242	30	

Amoxicillin	Alone	7.5 ± 2.121		0.199
	A+S	13.5 ± 4.949	80	
	C+A	10.52 ± 2.12	40.27	
	M+A	8.0 ± 1.414	6.67	
	O+A	10.5 ± 3.535	40	
	E+A	10.0 ± 2.828	33.33	
	G+A	16.0 ± 2.828	113.33	

Streptomycin	Alone	9.5 ± 0.707		0.402
	A+S	13.5 ± 4.949	42.10	
	C+S	9.0 ± 1.414	-5.26	
	M+S	7.5 ± 2.121	-21.05	
	O+S	13.0 ± 4.242	36.84	
	E+S	9.0 ± 1.414	-5.26	
	G+S	13.0 ± 4.242	36.84	

M = metronidazole; O = oxytetracycline; A = amoxicillin; S = streptomycin; G = gentamicin; C=co-amoxiclav; E = enrofloxacin.

**Table 4:** Synergy testing of drugs against methicillin-resistant *Staphylococcus aureus.*

Combinations	MIC AB	MIC A	FIC A	MIC BA	MIC B	FIC B	FICI	Results
amoxi+co-amoxiclav	5.86	11.72	0.5	1.95	5.86	0.33	0.83	Additive
amoxi+metro	15.62	11.72	1.33	250	375	0.67	2	Indifferent
amoxi+enro	4.56	11.72	0.39	0.98	1.95	0.5	0.89	Additive
amoxi+strepto	3.91	11.72	0.33	7.81	15.62	0.5	0.83	Additive
amoxi+genta	2.93	11.72	0.25	0.98	3.91	0.25	0.5	Synergistic
amoxi+oxy	23.44	11.72	2	31.25	15.62	2	4	Antagonistic
co-amoxiclav+metro	4.56	5.86	0.78	125	375	0.33	1.11	Indifferent
co-amoxiclav+enro	2.93	5.86	0.5	0.49	1.95	0.25	0.75	Additive
co-amoxiclav+strepto	3.91	5.86	0.67	7.81	15.62	0.5	1.17	Indifferent
co-amoxiclav+genta	2.93	5.86	0.5	1.95	3.91	0.5	1	Additive
co-amoxiclav+oxy	15.62	5.86	2.67	62.5	15.62	4	6.67	Antagonistic
metro+enro	31.25	375	0.08	0.49	1.95	0.25	0.33	Synergistic
metro+strepto	125	375	0.33	15.62	15.62	1	1.33	Indifferent
metro+genta	187.5	375	0.5	1.95	3.91	0.5	1	Indifferent
metro+oxy	500	375	1.33	62.5	15.62	4	5.33	Antagonistic
enro+strepto	3.91	1.95	2	7.81	15.62	0.5	2.5	Indifferent
enro+genta	0.49	1.95	0.25	1.95	3.91	0.5	0.75	Additive
enro+oxy	7.81	1.95	4	7.81	15.62	0.5	4.5	Antagonistic
strepto+genta	5.86	15.62	0.37	4.56	3.91	1.17	1.55	Indifferent
strepto+oxy	20.51	15.62	1.31	18.23	15.62	1.17	2.48	Indifferent
genta+oxy	7.81	3.91	2	20.51	15.62	1.31	3.31	Indifferent

co-amoxiclav = co-amoxiclav; enro = enrofloxacin; metro = metronidazole; genta = gentamicin; oxy = oxytetracycline; amoxi = amoxicillin; strepto = streptomycin.

## Data Availability

Supplementary file is attached for some of the data related to this article.

## Supplementary Materials

Supplementary Materials Supplementary Table 1: drug combinations and dosage regimens. Supplementary Table 2: *S. aureus* thermal nuclease protein conserved domain structure (reference sequence, Staph-1, Staph-2, and Staph-3). Supplementary Figure 1: multiple sequence alignment of *S. aureus Nuc* gene (reference and local isolate PK nucleotide sequences). Supplementary Figure 2: motif locations in gene sequences (1 to 5), sequence of individual motif and *p* value of motifs in sequences 1 to 5. Supplementary Figure 3: structural analysis of *S. aureus Nuc* gene from Pakistan. Supplementary Figure 4: antibacterial activity of different antibiotics/drugs against *S. aureus* (i) disc diffusion assay (1 = chloramphenicol; 2 = linezolid; 3 = levofloxacin; 4 = gentamicin; 5 = vancomycin), (ii) well diffusion assay (1 = metronidazole; 2 = co-amoxiclav; 3 = enrofloxacin; 4 = co-amoxiclav+metronidazole; 5 = enrofloxacin+metronidazole; 6 = co-amoxiclav+enrofloxacin; 7 = gentamicin).
